The article "Evaluating polymicrobial immune responses in patients suffering from tick-borne diseases" was retracted in 2022. Reasons: unreliable results or conclusions; concerns about the data.

# Evaluating polymicrobial immune responses in patients suffering from tick-borne diseases

**DOI:** 10.1038/s41598-018-34393-9

**Published:** 2018-10-29

**Authors:** Kunal Garg, Leena Meriläinen, Ole Franz, Heidi Pirttinen, Marco Quevedo-Diaz, Stephen Croucher, Leona Gilbert

**Affiliations:** 1 Department of Biological and Environmental Sciences, NanoScience Center, University of Jyväskylä, Jyväskylä, Finland; 2 Te?ted Ltd, Mattilaniemi 6-8, Jyväskylä, Finland; 3 Institute of Virology, Biomedical Research Center, Slovak Academy of Sciences, Bratislava, Slovak Republic; 4 School of Communication, Journalism, and Marketing, Massey University, Wellington, New Zealand

## Abstract

There is insufficient evidence to support screening of various tick-borne diseases (TBD) related microbes alongside Borrelia in patients suffering from TBD. To evaluate the involvement of multiple microbial immune responses in patients experiencing TBD we utilized enzyme-linked immunosorbent assay. Four hundred and thirty-two human serum samples organized into seven categories followed Centers for Disease Control and Prevention two-tier Lyme disease (LD) diagnosis guidelines and Infectious Disease Society of America guidelines for post-treatment Lyme disease syndrome. All patient categories were tested for their immunoglobulin M (IgM) and G (IgG) responses against 20 microbes associated with TBD. Our findings recognize that microbial infections in patients suffering from TBDs do not follow the one microbe, one disease Germ Theory as 65% of the TBD patients produce immune responses to various microbes. We have established a causal association between TBD patients and TBD associated co-infections and essential opportunistic microbes following Bradford Hill’s criteria. This study indicated an 85% probability that a randomly selected TBD patient will respond to Borrelia and other related TBD microbes rather than to Borrelia alone. A paradigm shift is required in current healthcare policies to diagnose TBD so that patients can get tested and treated even for opportunistic infections.

## Introduction

Tick-borne diseases (TBDs) have become a global public health challenge and will affect over 35% of the global population by 2050^1^. The most common tick-borne bacteria are from the *Borrelia burgdorferi sensu lato* (*s*.*l*.) group. However, ticks can also transmit co-infections like *Babesia* spp.^2^, *Bartonella* spp.^3^, *Brucella* spp.^4–8^, *Ehrlichia* spp.^9^, *Rickettsia* spp.^10,11^, and tick-borne encephalitis virus^12–14^. In Europe and North America, 4–60% of patients with Lyme disease (LD) were co-infected with *Babesia*, *Anaplasma*, or *Rickettsia*^11,15,16^. Evidence from mouse and human studies indicate that pathogenesis by various tick-borne associated microbes^15–17^ may cause immune dysfunction and alter, enhance the severity, or suppress the course of infection due to the increased microbial burden^18–22^. As a consequence of extensive exposure to tick-borne infections^15–17^, patients may develop a weakened immune system^22,23^, and present evidence of opportunistic infections such as *Chlamydia* spp.^24–27^, Coxsackievirus^28^, Cytomegalovirus^29^, Epstein-Barr virus^27,29^, Human parvovirus B19^24^, and *Mycoplasma* spp.^30,31^. In addition to tick-borne co-infections and non-tick-borne opportunistic infections, pleomorphic Borrelia persistent forms may induce distinct immune responses in patients by having different antigenic properties compared to typical spirochetes^32–35^. Nonetheless, current LD diagnostic tools do not include Borrelia persistent forms, tick-borne co-infections, and non-tick-borne opportunistic infections.

The article "Evaluating polymicrobial immune responses in patients suffering from tick-borne diseases" was retracted in 2022. Reasons: unreliable results or conclusions; concerns about the data.

The two-tier guidelines^36–38^ for diagnosing LD by the Centers for Disease Control and Prevention (CDC) have been challenged due to the omission of co-infections and non-tick-borne opportunistic infections crucial for comprehensive diagnosis and treatment^39,40^. Emerging diagnostic solutions have demonstrated the usefulness of multiplex assays to test for LD and tick-borne co-infections^41,42^. However, these new technologies do not address seroprevalence of non-tick-borne opportunistic infections in patients suffering from TBD and they are limited to certain co-infections^41,42^. Non-tick-borne opportunistic microbes can manifest an array of symptoms^24,29^ concerning the heart, kidney, musculoskeletal, and the central nervous system as seen in patients with Lyme related carditis^43^, nephritis^44^, arthritis^45^, and neuropathy^46^, respectively. Therefore, *Chlamydia* spp., Coxsackievirus, Cytomegalovirus, Epstein-Barr virus, Human parvovirus B19, *Mycoplasma* spp., and other non-tick-borne opportunistic microbes play an important role in the differential diagnosis of LD^24,29^. As the current knowledge regarding non-tick-borne opportunistic microbes is limited to their use in differential diagnosis of LD, it is unclear if LD patients can present both tick-borne co-infections and non-tick-borne opportunistic infections simultaneously.

For the first time, we evaluate the involvement of Borrelia spirochetes, Borrelia persistent forms, tick-borne co-infections, and non-tick-borne opportunistic microbes together in patients suffering from different stages of TBD. To highlight the need for multiplex TBD assays in clinical laboratories, we utilized the Bradford Hill’s causal inference criteria^47^ to elucidate the likelihood and plausibility of TBD patients responding to multiple microbes rather than one microbe. The goal of this study is to advocate screening for various TBD microbes including non-tick-borne opportunistic microbes to decrease the rate of misdiagnosed or undiagnosed^48^ cases thereby increasing the health-related quality of life for the patients^39^, and ultimately influencing new treatment protocol for TBDs.

The article "Evaluating polymicrobial immune responses in patients suffering from tick-borne diseases" was retracted in 2022. Reasons: unreliable results or conclusions; concerns about the data.

## Results

Positive IgM and IgG responses by CDC defined acute, CDC late, CDC negative, PTLDS immunocompromised, and unspecific patients to 20 microbes associated with TBD (Fig. 1) were utilized to evaluate polymicrobial infections (Figs 2–4). Furthermore, IgM and IgG responses from healthy individuals and patients from the remaining six categories with previous test results (Fig. 1, Table S1) were included for receiver operating characteristics (ROC) and diagnostic performance assessments (Figs 5 and S4–S6).

**Figure 1:** Patient flow diagram. In total, 509 human serum samples were received from various clinical laboratories. Patient samples that arrived without information regarding TBD related symptoms, clinical test results or the diagnosis by a healthcare professional were excluded (*n* = 77). Remaining 432 patients were tested for their IgM and IgG responses against 20 microbes associated with TBDs. Further, included patients were organized into seven categories based on their respective clinical pictures that followed the Centers for Disease Control and Prevention (CDC) two-tier diagnosis guidelines for Lyme disease, Infectious Disease Society of America (IDSA) guidelines for Post-treatment Lyme Disease Syndrome (PTLDS), and literature regarding the use of lymphocyte and low CD57 cell count in diagnosing patients for Lyme disease. Patient categories included CDC acute (*n* = 43), CDC late (*n* = 43), CDC negative (*n* = 46), PTLDS (*n* = 31), immunocompromised (*n* = 61), unspecific (*n* = 31), and healthy (*n* = 177).

**Figure 2:** Polymicrobial infections are present at all stages of tick-borne diseases. (**A**) Overall positive immunoglobulin M (IgM), and immunoglobulin G (IgG) responses by patients to none, one, or multiple microbes. (**B**) Overall positive IgM and IgG reactions by patients to 20 individual microbes. (**C**) IgM and IgG responses by individual patient categories to 20 microbes. Patient categories refer to individuals from Centers for Disease Control and Prevention (CDC) acute, CDC late, CDC negative, Post-Treatment Lyme Disease Syndrome (PTLDS), immunocompromised, and unspecific. Additionally, only 2C includes IgM and IgG responses by healthy individuals to 20 microbes. Microbes include *Borrelia burgdorferi sensu stricto*, *Borrelia afzelii*, *Borrelia garinii*, *Borrelia burgdorferi sensu stricto* persistent form, *Borrelia afzelii* persistent form, *Borrelia garinii* persistent form, *Babesia microti*, *Bartonella henselae*, *Brucella abortus*, *Ehrlichia chaffeensis*, *Rickettsia akari*, Tick-borne encephalitis virus (TBEV), *Chlamydia pneumoniae*, *Chlamydia trachomatis*, Coxsackievirus A16 (CVA16), Cytomegalovirus (CMV), Epstein-Barr virus (EBV), *Mycoplasma pneumoniae*, *Mycoplasma fermentans*, and Human parvovirus B19 (HB19V).

The article "Evaluating polymicrobial immune responses in patients suffering from tick-borne diseases" was retracted in 2022. Reasons: unreliable results or conclusions; concerns about the data.

**Figure 3:** Lyme disease diagnostic tests should incorporate *Borrelia burgdorferi sensu stricto*, *Borrelia afzelii*, and *Borrelia garinii* in spirochetes and persistent forms. (**A** and **B**) immunoglobulin M (IgM) and immunoglobulin G (IgG) responses by patients to different forms of Borrelia and other TBD microbes. Patients refer to individuals from categories Centers for Disease Control and Prevention (CDC) acute, CDC late, CDC negative, Post-Treatment Lyme Disease Syndrome (PTLDS), immunocompromised, and unspecific. Other TBD microbes include *Babesia microti*, *Bartonella henselae*, *Brucella abortus*, *Ehrlichia chaffeensis*, *Rickettsia akari*, Tick-borne encephalitis virus (TBEV), *Chlamydia pneumoniae*, *Chlamydia trachomatis*, Coxsackievirus A16 (CVA16), Cytomegalovirus (CMV), Epstein-Barr virus (EBV), *Mycoplasma pneumoniae*, *Mycoplasma fermentans*, and Human parvovirus B19 (HB19V). (A.1 and B.1) Distribution of IgM and IgG levels to different species of Borrelia spirochetes and (A.2 and B.2) Borrelia persistent forms. Abbreviations Bb, Ba, and Bg depict *Borrelia burgdorferi sensu stricto*, *Borrelia afzelii*, and *Borrelia garinii*, respectively.

**Figure 4:** Response to Borrelia spirochetes and persistent forms increases reaction frequency to other TBD microbes. Immunoglobulin M (IgM) and immunoglobulin G (IgG) responses by patients (**A**) to different forms of Borrelia alone versus reactions to different forms of Borrelia together with other TBD microbes, (**B**) to the number of other TBD microbes with distinctive forms of Borrelia, and (**C**) to other specific TBD microbes together with different forms of Borrelia. Other TBD microbes include *Babesia microti*, *Bartonella henselae*, *Brucella abortus*, *Ehrlichia chaffeensis*, *Rickettsia akari*, Tick-borne encephalitis virus (TBEV), *Chlamydia pneumoniae*, *Chlamydia trachomatis*, Coxsackievirus A16 (CVA16), Cytomegalovirus (CMV), Epstein-Barr virus (EBV), *Mycoplasma pneumoniae*, *Mycoplasma fermentans*, and Human parvovirus B19 (HB19V).

**Figure 5:** Collective immunoglobulin M (IgM) and immunoglobulin G (IgG) responses should be considered for diagnosing Lyme disease. (**A**) IgM, IgG, and collective IgM/IgG nonparametric receiver operating characteristic (ROC) curves for different forms of Borrelia. AUC and 95% CI denote Area under the curve, and 95% confidence interval, respectively. (**B**) IgM, IgG, and collective IgM/IgG diagnostic performance characteristics for different forms of Borrelia represented with 95% confidence interval line across the marker. Borrelia species included in the analyses are *Borrelia burgdorferi sensu stricto*, *Borrelia afzelii*, and *Borrelia garinii*. IgM and IgG responses from healthy individuals and others with previous test results (Fig. 1, Table S2) were included for ROC and diagnostic performance assessments (Figs 5 and S4–S6).

The article "Evaluating polymicrobial immune responses in patients suffering from tick-borne diseases" was retracted in 2022. Reasons: unreliable results or conclusions; concerns about the data.

### Immune responses to multiple TBD associated microbes at all stages of TBDs

In Fig. 2A, 51% and 65% of patients had IgM and IgG responses to more than one microbe, whereas 9% and 16% of patients had IgM and IgG responses to only one microbe, respectively. On average, 23% and 31% of patients had IgM and IgG responses for each of the microbes, respectively (Fig. 2B). The Shapiro-Wilk test and Q-Q plot implied that patient responses to 20 microbes were normally distributed for IgM and IgG (Fig. S1). Immune responses to Borrelia persistent forms (all three species) for IgM and IgG were 5–10% higher compared to Borrelia spirochetes in all three species (Fig. 2B). Interestingly, the probability that a randomly selected patient will respond to Borrelia persistent forms rather than the Borrelia spirochetes (Fig. S2) is 80% (*d* = 1.2) for IgM and 68% for IgG (*d* = 0.7). Figure 2A and B indicated that IgM and IgG responses by patients from different stages of TBDs are not limited to only Borrelia spirochetes.

Patients from the seven categories demonstrated IgM and IgG responses to multiple microbes (Fig. 2C). On average, 32% and 23% of individuals from the CDC defined acute category had IgM and IgG responses to various microbes, respectively. In the CDC defined late category, the corresponding percentages were 31% and 44%. Surprisingly, about 13% of the CDC defined negative patients had IgM and 36% had IgG responses to different microbes. Remarkably, 72% of the CDC defined negative patients responded to at least one Borrelia species’ persistent form (Fig. S2). In the PTLDS category, the average percentage of individuals that responded to several microbes were 27% for IgM and 33% for IgG. The odds that a PTLDS patient at random will respond to Borrelia persistent forms rather than the Borrelia spirochetes are 76% (*d* = 1.0) for IgM and an astonishing 95% (*d* = 2.4) for IgG (Fig. S2). Furthermore, roughly 22% and 30% of individuals from the immunocompromised category had IgM and IgG responses to different microbes, respectively. For patients in the unspecific category, 12% had IgM and 18% had IgG responses to multiple microbes. In addition, the two-tailed Fisher’s exact test revealed that 90% of IgM responses and 97.5% of the IgG responses to 20 microbes (Table 1) by patients from CDC defined acute, CDC late, CDC negative, PTLDS, immunocompromised and unspecific categories were statistically different (i.e., *p* ≤ 0.05) from healthy individuals (Fig. S3). Results from Fig. 2C suggested that polymicrobial infections in these patients are not limited to a particular stage of TBD.

The article "Evaluating polymicrobial immune responses in patients suffering from tick-borne diseases" was retracted in 2022. Reasons: unreliable results or conclusions; concerns about the data.

**Table 1:** List of microbial antigens and their types included in this study.

Microbial antigen	Antigen type	References
*Borrelia burgdorferi sensu stricto*	Lysate	^33^
*Borrelia afzelii*	Lysate	
*Borrelia garinii*	Lysate	
*Borrelia burgdorferi sensu stricto* persistent form	Lysate	
*Borrelia afzelii* persistent form	Lysate	
*Borrelia garinii* persistent form	Lysate	
*Babesia microti*	Peptide	^101^
*Bartonella henselae*	Peptide	^102^
*Brucella abortus*	Peptide	^103^
*Ehrlichia chaffeensis*	Peptide	^101^
*Rickettsia akari*	Lysate	^104^
Tick-borne encephalitis virus	Peptide	^105^
*Chlamydia pneumoniae*	Peptide	^106^
*Chlamydia trachomatis*	Peptide	^107^
Coxsackievirus A16	Peptide	^108^
Cytomegalovirus	Peptide	^109^
Epstein-Barr virus	Peptide	^110^
Human parvovirus B19	Peptide	^111, 112^
*Mycoplasma pneumoniae*	Peptide	^113^
*Mycoplasma fermentans*	Peptide	^114^

### Immune reponses to multiple species of Borrelia spirochetes and persistent forms

In Fig. 3, 26% of the patients presented an IgM response to both spirochetes and persistent forms whereas only 2% responded to spirochetes and 13% to persistent forms alone. Similarly, 39% of the patients had an IgG response to both spirochetes and persistent forms compared to 7% and 13% that responded to only the spirochetes or persistent forms, respectively. It was noted that 40% and 20% of the patients did not produce an IgM and IgG response, respectively against Borrelia spirochete and the persistent forms (Table 1). Figure 3 sub-inlets (Fig. 3A.1, A.2, B.1 and B.2) indicate individual strains of Borrelia that the patients were responding to in the initial category (i.e. spirochetes or persistent forms alone). In Fig. 3 sub-inlets, more than 50% of the patients reacted to only the individual Borrelia strains suggesting that Borrelia antigens are not cross-reactive. If patients were cross-reacting among antigens, a larger percentage of the patients would be seen with the combination of all three species (Fig. S2). These results provide evidence to suggest that the inclusion of different Borrelia species and their morphologies in current LD diagnostic tools will improve its efficiency.

The article "Evaluating polymicrobial immune responses in patients suffering from tick-borne diseases" was retracted in 2022. Reasons: unreliable results or conclusions; concerns about the data.

### Immune responses to Borrelia and TBD related microbes versus immune responses to only Borrelia

The difference in percentages of patients responding to only Borrelia (8% for IgM, and 12% for IgG) compared to patients responding to Borrelia and many other TBD microbes (61% for IgM and IgG) was great (Fig. 4A). The probability that a randomly selected patient will respond to Borrelia and other TBD microbes rather than to only Borrelia is 88% (*d* = 1.7) for IgM and 83% (*d* = 1.4) for IgG (Fig. S2). Moreover, the highest percentage of IgM (42%) and IgG (43%) responses against other TBD microbes was demonstrated in patients that responded to both Borrelia spirochetes and persistent forms (Fig. 4A). These patients also had antibodies against the highest number (14 other TBD microbes) of other TBD microbes (Fig. 4B). On average, 70% of the patients demonstrated IgM and IgG antibodies to other specific TBD microbes together with spirochetes and persistent forms (Fig. 4C). Outstandingly large immune responses to many other microbes and Borrelia signified the profound polymicrobial nature of tick-borne diseases (Fig. 4).

### Clinical sensitivity and specificity

The coefficients of intra and inter-assay variations of these ELISA assays were 4.5% and 15%, respectively. Further, a minimum 0.875 area under the receiver operating characteristic (ROC) curve (AUC) and *p* values < 0.001 were recorded for all forms of Borrelia in IgM, IgG, and collective IgM/IgG analyses (Fig. 5A). Interestingly, the collective IgM/IgG ROC curves demonstrated the largest AUC values (max 0.961) compared to AUC values from only IgM (max 0.885) or IgG (max 0.920) ROC curves. AUC values closer to 1 and *p* values < 0.001 suggest that the test protocol can effectively distinguish between healthy individuals and LD patients, especially when collective IgM/IgG reactions are considered (Fig. 5B). Collective IgM/IgG responses offer the highest sensitivity (max 94%) compared to sensitivity values from only IgM (max 64%) or IgG (max 88%). Similarly, the highest PPV (max 74%) was noted for collective IgM/IgG responses compared to only IgM (max 70%) or IgG (max 72%). However, for the different forms of Borrelia, the difference in specificity (91 ± 4%) or NPV (95 ± 3%) among IgM, IgG, and collective IgM/IgG was minute. Figure 5 recommends utilization of collective IgM/IgG responses to diagnose LD.

The collective IgM/IgG responses for all TBD associated co-infections and opportunistic infections exhibited largest AUC values. In Figs S4 and S5, AUC values for collective IgM/IgG responses ranged from 0.924 to 0.998. Also, AUC values for only IgM ranged from 0.787 to 0.933, and for IgG from 0.769 to 0.975. For tick-borne associated co-infections, the sensitivity ranged from 80% for *B*. *henselae* with 100% PPV, 93% for *E*. *chaffeensis* with 68% PPV, to 100% for *B*. *microti* with 13% PPV (Fig. S6). Likewise, the specificity extended from 94% for *B*. *microti* with 100% NPV, 97% for *E*. *chaffeensis* with 99% NPV, to 100% for *B*. *henselae* with 99% NPV (Fig. S6). In the case of tick-borne associated opportunistic microbes, the sensitivity ranged from 83% for CMV with 71% PPV, 88% for *C*. *trachomatis* with 58% PPV, 91% for EBV with 83% PPV, 91% for *M*. *pneumoniae* with 83% PPV, 92% for CVA16 with 92% PPV, to 93% for *C*. *pneumoniae* with 91% PPV (Fig. S6). Additionally, the specificity stretched from 97% for *C*. *trachomatis* with 99% NPV, 98% for *C*. *pneumoniae* with 98% NPV, 98% for EBV with 98% NPV, 98% for *M*. *pneumoniae* with 99% NPV, to 99% for CVA16 with 99% NPV, and 99% for CMV with 99% NPV (Fig. S6).

The article "Evaluating polymicrobial immune responses in patients suffering from tick-borne diseases" was retracted in 2022. Reasons: unreliable results or conclusions; concerns about the data.

## Discussions

To evaluate the involvement of polymicrobial infections in TBD, 432 patients diagnosed at different TBD stages were tested for their IgM and IgG immune responses to 20 microbes associated with TBDs (Fig. 1). The study outcome indicated that polymicrobial infections existed at all stages of TBD with IgM and IgG responses to several microbes (Fig. 2). Additionally, IgM and IgG responses to multiple TBD associated co-infections and opportunistic infections were large in patients that reacted to Borrelia compared to patients with no reaction to Borrelia (Fig. 4). However, on average 20% patients responded (IgM and IgG) to only TBD associated co-infections and opportunistic infections that demonstrates the importance of other TBD microbes in addition to Borrelia (Fig. 3). Results presented in this study propose that infections in patients suffering from TBDs do not obey the one microbe one disease Germ Theory. Based on these results and substantial literature^11,15–17,27,49–51^ on polymicrobial infections in TBD patients, we examined the probability of a causal relationship between TBD patients and polymicrobial infections following Hill’s nine criteria^47^.

An average effect size of *d* = 1.5 for IgM and IgG (Fig. 4A) responses is considered very large^52^. According to common language effect size statistics^53^, *d* = 1.5 indicates 85% probability that a randomly selected patient will respond to Borrelia and other TBD microbes rather than to only Borrelia. Reports from countries such as Australia^27^, Germany^49^, Netherlands^11^, Sweden^50^, the United Kingdom^51^, the USA^15,16^, and others indicate that 4% to 60% of patients suffer from LD and other microbes such as *Babesia microti* and human granulocytic anaplasmosis (HGA). However, previous findings^11,15,16,27,49–51^ are limited to co-infections (i.e., Babesia, Bartonella, Ehrlichia, or Rickettsia species) in patients experiencing a particular stage of LD (such as Erythema migrans). In contrast, a broader spectrum of persistent, co-infections, and opportunistic infections associated with diverse stages of TBD patients have been demonstrated in this study (Fig. 2). From a clinical standpoint, the likelihood for IgM and IgG immune responses by TBD patients to the Borrelia spirochetes versus the Borrelia persistent forms, and responses to just Borrelia versus Borrelia with many other TBD microbes has been quantified for the first time (Fig. S2).

The article "Evaluating polymicrobial immune responses in patients suffering from tick-borne diseases" was retracted in 2022. Reasons: unreliable results or conclusions; concerns about the data.

Borrelia pathogenesis could predispose individuals to polymicrobial infections because it can suppress, subvert, or modulate the host’s immune system^18–22^ to create a niche for colonization by other microbes^54^. Evidence in animals^55^ and humans^11,15,16,27,49–51^ frequently indicate co-existence of Borrelia with other TBD associated infections. Interestingly, IgM and IgG immune levels by patients to multiple forms of Borrelia resulted in immune responses to 14 other TBD microbes (Fig. 4B). In contrast, patient responses to either form of Borrelia (spirochetes or persistent forms) resulted in reactions to an average of 8 other TBD microbes (Fig. 4B). Reaction to two forms of Borrelia reflected an increase in disease severity indicating biological gradient for causation as required by Hill’s criteria^47^.

Multiple microbial infections in TBD patients seem plausible because ticks can carry more than eight different microbes depending on tick species and geography^56,57^. Moreover, Qiu and colleagues reported the presence of at least 18 bacterial genera shared among three different tick species and up to 127 bacterial genera in *Ixodes persulcatus*^58^. Interestingly, research indicates Chlamydia-like organism in *Ixodes ricinus* ticks and human skin^59^ that may explain immune responses to Chlamydia spp., seen in this study (Fig. 2). Additionally, prevalence of TBD associated co-infections such as *B*. *abortus*, *E*. *chaffeensis*, and opportunistic microbes such as *C*. *pneumoniae*, *C*. *trachomatis*, Cytomegalovirus, Epstein-Barr virus, and *M*. *pneumoniae* have been recorded in the general population of Europe and the USA (Table S2). However, true incidence of these microbes is likely to be higher considering underreporting due to asymptomatic infections and differences in diagnostic practices and surveillance systems across Europe and in the USA. More importantly, clinical evidence for multiple microbes has been reported in humans^11,15,16,27,49–51^, and livestock^55^ to mention the least. Our findings regarding the presence of polymicrobial infections at all stages of TBD further supports the causal relationship between TBD patients and polymicrobial infections (Fig. 2). Various microbial infections in TBD patients have been linked to the reduced health-related quality of life (HRQoL) and increased disease severity^39^.

The article "Evaluating polymicrobial immune responses in patients suffering from tick-borne diseases" was retracted in 2022. Reasons: unreliable results or conclusions; concerns about the data.

An association between multiple infections and TBD patients relates well to other diseases such as periodontal, and respiratory tract diseases. Oral cavities may contain viruses and 500 different bacterial species^60^. Our findings demonstrate that TBD patients may suffer from multiple bacterial and viral infections (Fig. 4). In respiratory tract diseases, influenza virus can stimulate immunosuppression and predispose patients to bacterial infections causing an increase in disease severity^61^. Likewise, Borrelia can induce immunosuppression that may predispose patients to other microbial infections causing an increase in disease severity.

Traditionally, positive IgM immune reaction implies an acute infection, and IgG response portrays a dissemination, persistent or memory immunity due to past infections. Depending on when TBD patients seek medical advice, the level of anti-Borrelia antibodies can greatly vary as an Erythema migrans (EM) develops and may present with IgM, IgG, collective IgM/IgG, or IgA^62^. This study recommends both IgM and IgG in diagnosing TBD (Figs 5 and S4–S6) as unconventional antibody profiles have been portrayed in TBD patients. Presence of long-term IgM and IgG antibodies have been reported in LD patients that were tested by the CDC two-tier system. In 2001, Kalish and colleagues reported anti-Borrelia IgM or IgG persistence in patients that suffered from LD 10–20 years ago^63^. Similarly, Hilton and co-workers recorded persistent anti-Borrelia IgM response in 97% of late LD patients that were considered cured following an antibiotic treatment^64^.

Similar events of persistent IgM and IgG antibody reactions were demonstrated in patients treated for Borrelia arthritis and acrodermatitis chronica atrophicans^65^, chronic cutaneous borreliosis^66^, and Lyme neuroborreliosis^67^. A clear phenomenon of immune dysfunction is occurring, which might account for the disparities in LD patient’s antibody profiles and persistence. Borrelia suppresses the immune system by inhibition of antigen-induced lymphocyte proliferation^18^, reducing Langerhans cells by downregulation of major histocompatibility complex class II molecules on these cells^19^, stimulating the production of interleukin-10 and anti-inflammatory immunosuppressive cytokine^20^, and causing disparity in regulation and secretion of cytokines^21^. Other studies have demonstrated low production or subversion of specific anti-Borrelia antibodies in patients with immune deficiency status^22^.

The article "Evaluating polymicrobial immune responses in patients suffering from tick-borne diseases" was retracted in 2022. Reasons: unreliable results or conclusions; concerns about the data.

Following Hill’s nine criteria^47^ a causal association between TBD patients and polymicrobial infections can be established because the likelihood (Fig. S2F) of TBD patients responding to Borrelia and various other TBD microbes is substantial (strength of association). Evidence concerning immune responses to multiple forms of Borrelia and 14 other TBD microbes versus responses to either type of Borrelia and 8 other TBD microbes (Fig. 4B) explains Hill’s biological gradient criteria. Also, immune responses to several microbes at all stages of TBD (Fig. 2C) and the large difference in immune responses (Fig. 4A) by individuals to only Borrelia (10%) and Borrelia with many other TBD microbes (60%) realize Hill’s specificity and experimental evidence standards. Former studies that reveal tick microbiome can contain various microbes^56,58^, co-infections in LD patients from multiple countries^11,15,16,27,49–51^, and the ability of Borrelia to manipulate its host’s immune system to promote colonization by other microbes^18–22,54^ meet Hill’s plausibility, consistency, temporality, and coherence of association conditions. Finally, the role of polymicrobial infections in periodontal^60^, respiratory tract^61^, and other diseases fulfil Hill’s analogy criteria.

Our study has several limitations. First, commercial laboratories that contributed samples to our study had strict policies for patient de-identification and data protection. Thus, the demographic information such as age, sex, region and ethnicity relating to many patients included in this study are missing. Second, all Cohen’s *d* effect size analyses (Fig. S2) included in this study were substantively significant (Cohen’s *d*) but not statistically noteworthy (*t* statistic). However, the statistically non-significant effect size is not futile because unlike the *t* statistic, Cohen’s *d* is independent of sample variability and size^52,68^.

In the USA alone, the economic healthcare burden for patients suffering from LD and ongoing symptoms is estimated to be $1.3 billion per year^69^. Additionally, 83% of all TBD diagnostic tests performed by the commercial laboratories in the USA accounted for only LD^70^. Globally, the commercial laboratories’ ability to diagnose LD has increased by merely 4% (weighted mean for ELISA sensitivity 62.3%) in the last 20 years^71^. This study provides evidence regarding polymicrobial infections in patients suffering from different stages of TBDs. Literature analyses and results from this study followed Hill’s criteria indicating a causal association between TBD patients and polymicrobial infections. Also, the study outcomes indicate that patients may not adhere to traditional IgM and IgG responses.

The article "Evaluating polymicrobial immune responses in patients suffering from tick-borne diseases" was retracted in 2022. Reasons: unreliable results or conclusions; concerns about the data.

## Materials and Methods

### Ethics statement

Left over and disregarded human sera collected was approved by the Federal Institute for Drugs and Medical Devices, Germany (project no. 95.10-5661-7066); and Western Institutional Review Board, United States of America (USA) (USMA201441, WIRB® protocol #20141439). Demographic information concerning age, sex, and ethnicity of the patients was not provided for all sera samples included in this study due to the strict patient de-identification and data protection policies followed by contributing commercial laboratories. Sera samples that were provided with patient’s demographic information comprised adults and child participants. Written and informed consent was obtained from all patients enrolled in this study. In the case of child participants, written and informed consent was obtained either from a parent or a guardian. All methods were performed in accordance with relevant guidelines and regulations.

### Study design

Immunoglobulin M (IgM) and G (IgG) levels of all eligible patients (Fig. 1) were tested on an enzyme-linked immunosorbent assay (ELISA) against 20 microbial antigens (Table 1). Antigen selection included lysates or peptides for Borrelia and TBD associated co-infections and opportunistic infections (latter hereon collectively referred to as other TBD microbes). To evaluate polymicrobial infections in patients suffering from different stages of TBDs, patients were organized into seven categories according to their respective clinical diagnosis provided by healthcare professionals (Fig. 1).

### Human serum sample collection and categorization

Between May 2014 and September 2016, 509 human serum samples were received from clinical laboratories in Europe and the United States. Samples that arrived without information regarding TBD related symptoms, clinical test results or the diagnosis by a healthcare professional were excluded (Fig. 1). The remaining 432 patients (completion rate of 85%) were tested for their IgM and IgG responses against 20 microbes associated with TBDs (Table 1). Among the 432 patients, 347 (i.e., 80%) specimens were received from clinical laboratories and medical doctors across Europe. Likewise, remaining 85 (i.e., 20%) sera samples were collected from clinical laboratories and medical doctors in the United States. Several sera samples included commercial diagnosis for other TBD microbes (Table S1). Eligible patients were organized into seven categories according to their respective clinical diagnosis as follows.

1. CDC acute (*n* = 43). Patients suffered from flu-like symptoms, presented an EM rash, and tested positive for IgM serology utilizing Centers for Disease Control and Prevention (CDC) two-tier Lyme disease (LD) diagnosis criteria^36–38^.
2. CDC late (*n* = 43). Patients suffered from late LD symptoms (a headache, arthritic pain, joint pain, etc.) and tested positive for IgG serology utilizing CDC two-tier LD diagnosis criteria^36–38^. Also, patients suffered from CDC approved late LD symptoms such as Lyme arthritis, carditis, or neurological symptoms that included sure signs and symptoms involving the heart, joints, peripheral or central nervous system^37,72^.
3. CDC negative (*n* = 46). Patients suffered from a combination of flu-like symptoms and late LD symptoms but tested negative for IgM and IgG serology utilizing the CDC two-tier LD diagnosis criteria^36–38^.
4. Post-treatment Lyme disease syndrome [PTLDS (*n* = 31)]. Patients were diagnosed with PTLDS by Lyme Literate Medical doctors according to the Infectious Disease Society of America (IDSA) guidelines^73,74^.
5. Immunocompromised (*n* = 61). Patients suffered from a combination of flu-like symptoms and late LD symptoms^36–38^. Patients were tested for low CD57 cell count and a negative immune response by lymphocyte cells to Borrelia antigens. Rational here is that if CD57 cell count is low, then the patient would be persistent or progressive with LD^75–77^.
6. Unspecific (*n* = 31). Patients suffered from a combination of flu-like symptoms and late LD that followed CDC two-tier LD diagnosis criteria^36–38^. However, no test results were provided to support and reason with the documented symptoms. Thus, the category was termed as “unspecific”.
7. Healthy (*n* = 177) for each antibody type (77 for IgM, 77 for IgG, and 23 for both IgM and IgG). Individuals did not suffer from any combination of flu-like symptoms and late LD symptoms^36–38^. Healthy individuals tested negative for IgM and IgG serology utilizing the CDC two-tier LD diagnosis criteria^36–38^. Also, healthy blood donors were included.

The article "Evaluating polymicrobial immune responses in patients suffering from tick-borne diseases" was retracted in 2022. Reasons: unreliable results or conclusions; concerns about the data.

### Enzyme-linked immunosorbent assay (ELISA) procedure

All microbial peptides (Table 1) were synthesized at >95% purity by GeneCust, Luxembourg. High Performance Liquid Chromatography and Mass Spectrometry were utilized by GeneCust to ensure specified peptide quality. The protein concentrations of cell lysates were measured with ND 1000 spectrophotometer (Finnzymes) at 280 nm. Fresh antigen stock solutions (1 mg/ml) were diluted at 1:100 in 0.1 M carbonate buffer (0.1 M Na_2_CO_3_/0.1 M NaHCO_3_, pH 9.5). Dilution volume was equally divided among stock solutions for microbes with two peptide sequences. Human IgM (Sigma) and human IgG (Sigma) were utilized as positive controls in this study. Additionally, human IgM and human IgG were interchangeably used as negative control for each other. The control stock solutions were diluted similarly as antigens.

Flat bottom 96-well polystyrene ELISA plates (Nunc) were coated with 100 µl of antigens and controls as duplicates and incubated at 4 °C overnight. Post incubation, the plates were washed three times with 300 µl of PBS-Tween (PBS + 0.05% Tween 20) using DNX-9620G (Nanjing Perlove Medical Equipment Co., Ltd) microplate washer and were then coated with 100 µl of 2% BSA (Sigma) in PBS. After an overnight incubation at 4 °C, the 2% BSA in PBS was discarded. Further, 100 µl of patient serum diluted at 1:200 in 1% BSA/PBS was added. The plates were then allowed to incubate for 2 hrs at room temperature (RT). Post incubation, the plates were washed five times with 300 µl of PBS-Tween. An amount of 100 µl of Horse Radish Peroxidase (HRP) conjugated to mouse anti-human IgG (Abcam) or rabbit anti-human IgM (Antibodies Online) was introduced to the plates at 1:10000 or 1:1000 dilution factor, respectively. After 1.5 hr incubation at RT, the plates were washed five times with 300 µl of PBS-Tween and were then supplemented with 100 µl of 3,3′,5,5′ tetramethylbenzidine substrate (TMB, Thermo-Pierce). Plates containing HRP conjugated to mouse anti-human IgG or IgM were incubated at RT for 5 min or 1 hr, respectively. The catalytic reaction between anti-human antibodies and TMB substrate was stopped by adding 100 µl of 2 M H_2_SO_4_. Victor^TM^ X4 multi-label plate reader (Perkin Elmer) was utilized to measure the optical density (OD) values at 450 nm at 0.1 sec.

### ELISA data compilation for statistical and graphical analyses

Duplicate OD values for each antigen were assessed to be within 30% range of each other^78–81^. To establish cut-off values for IgM and IgG of each antigen, values from healthy category were used. Cut-off values were established by adding mean of all average OD values to three times the standard deviation of all average OD values^79,80^. In the next step, an optical density index (ODI) dataset was created for all patient categories by dividing average OD values of microbes by their respective cut-off values. Finally, ODI values ≤ 0.8, 0.8 ≤ 0.99, and ≥1 were coded as 0, 2, and 1, respectively. ODI values ≤ 0.8, 0.8 ≤ 0.99, and ≥1 represent negative, borderline, and positive immune responses by patients, respectively. For all antigens, borderline responses were combined with positive results^82^ because literature is rife with evidence regarding immune dysfunction in TBD patients^62–67,83–91^. In all graphical analyses, IgM and IgG responses to *Borrelia burgdorferi sensu stricto*, *Borrelia afzelii*, and *Borrelia garinii* were grouped as spirochetes. To *Borrelia burgdorferi sensu stricto*, *Borrelia afzelii*, and *Borrelia garinii* persistent forms were grouped as persistent forms. Responses to the three species for Borrelia and their different morphological forms were grouped as spirochetes and persistent forms. Finally, patients with IgM and IgG response to only other TBD microbes and not Borrelia were grouped.

The article "Evaluating polymicrobial immune responses in patients suffering from tick-borne diseases" was retracted in 2022. Reasons: unreliable results or conclusions; concerns about the data.

### Statistical analyses

To validate positive patient response distribution curve among 20 microbes, Shapiro-Wilk test^92^ was computed using SPSS. Shapiro-Wilk test results were verified using the normal Q-Q plot for IgM and IgG^92^. Cohen’s *d*^52,93^ effect size with 95% confidence interval (CI)^94^ was calculated to measure the strength of association and probability of superiority among various experimental and control groups such as patients that responded to Borrelia and multiple other TBD microbes (experimental group) versus patients that responded to only Borrelia (control group). An effect size of *d* ≥ 0.2, *d* ≥ 0.5, *d* ≥ 0.8, and *d* ≥ 1 was considered small, medium, large, and very large, respectively^52,93^. For each Cohen’s *d* estimation, a two-tailed *t*-test assuming unequal variance among the experimental and control groups was performed^95^. The *t*-test results *p* ≤ 0.05 were considered statistically significant^95^. Two-tailed Fisher’s exact test was used to assess if the IgM and IgG responses to 20 microbes (Table 1) by patients from the CDC defined acute, CDC late, CDC negative, PTLDS, immunocompromised, and unspecific categories were statistically different (i.e., *p* ≤ 0.05) compared to healthy individuals. GraphPad Software was utilized to perform the two-tailed Fisher’s exact test. The coefficient of variation (CV) was assessed by calculating intra- and inter-assay variation^96^. Intra-assay variation was determined by a duplicate high titer and low titer measurement from the same plate. For inter-assay, variation was determined by measuring six high titer samples and six low titer samples from different plates that were performed on different days by different operators.

Nonparametric receiver operating characteristic (ROC) curves were created in SPSS^97–99^ to evaluate the diagnostic assay’s ability to discriminate between healthy individuals and TBD patients. Parameters to understand ROC curves included area under the curve (AUC) with 95% CI^100^, and *p* values (*p* < 0.05 were interpreted significant)^97–99^. Diagnostic performance characteristics for each antigen such as sensitivity, specificity, positive predictive value (PPV), and negative predictive value (NPV) with 95% CI^100^ were calculated by a corresponding previous clinical diagnosis of patients with ELISA results from this study. MEDCALC^®^ was utilized for calculating performance characteristics. ROC curves and performance characteristics for *Brucella abortus*, *Rickettsia akari*, Tick-borne encephalitis virus, Human parvovirus B19, and *Mycoplasma fermentans* were not calculated due to insufficient clinical data. ROC curves and diagnostic performance parameters were analyzed for IgM, IgG, and collective IgM/IgG responses. For collective IgM/IgG analyses, positive or borderline response to an antigen in either IgM or IgG was considered positive. A negative response to an antigen in both IgM and IgG was regarded as negative.

The article "Evaluating polymicrobial immune responses in patients suffering from tick-borne diseases" was retracted in 2022. Reasons: unreliable results or conclusions; concerns about the data.

### Causal inference and epidemiology search strategy

This study attempts to establish a causal relationship between TBD patients and multiple microbial infections following Bradford Hill’s nine criteria that includes strength, consistency, specificity, temporality, biological gradient, plausibility, coherence, experiment, and analogy^47^. Strength requires a statistically significant association between TBD patients and multiple microbial infections. In the next step, literature was obtained from various countries concerning polymicrobial infections in TBD patients that will fulfil the consistency, plausibility, and coherence criteria. IgM or IgG immune responses by TBD patients to many microbes (Table 1) in the presence of an immune response to a specific or group of microbes will confirm the specificity and experiment criteria. Further, to prove temporality, it is essential to understand if those particular microbes can dispose TBD patients to multiple microbial infections. An increase in IgM or IgG response to microbes that confirm Hill’s specificity should also boost response to many microbes to display biological gradient. Lastly, evidence concerning multiple microbial infections in diseases other than TBD will fulfil the analogy criteria.

CDC and European CDC (ECDC) reports were utilized to review the incidence rate per 100,000 population in U.S.A. and Europe for TBD associated co-infections and opportunistic microbes (Table 1). In cases where CDC or ECDC reports were unavailable, PubMed and Google Scholar assisted. The search query used in PubMed and Google Scholar included a name for the microbe followed by the phrase “incidence rate and U.S.A.” or “incidence rate and Europe”; for example, Babesia microti incidence rate and U.S.A. or Babesia microti incidence rate and Europe (Table S2).

The article "Evaluating polymicrobial immune responses in patients suffering from tick-borne diseases" was retracted in 2022. Reasons: unreliable results or conclusions; concerns about the data.

## Electronic supplementary material

Supplementary information file

## Data Availability

All data generated or analysed during this study are included in this published article (see supplementary information file).
